# Fingolimod Nanoemulsions at Different Particle Sizes Define the Fate of Spinal Cord Injury Recovery

**DOI:** 10.1155/2022/5703426

**Published:** 2022-08-16

**Authors:** Delaram Poormoghadam, Bita Rasoulian Shiadeh, Fereshte Azedi, Hani Tavakol, Seyed Mahdi Rezayat, Shima Tavakol

**Affiliations:** ^1^University of Amsterdam, Amsterdam, Netherlands; ^2^School of Biomedical Sciences, Vrije Universiteit Amsterdam, Amsterdam, Netherlands; ^3^Cellular and Molecular Research Center, Iran University of Medical Sciences, Tehran, Iran; ^4^Department of Neuroscience, Faculty of Advanced Technologies in Medicine, Iran University of Medical Sciences, Tehran, Iran; ^5^Department of Medical Nanotechnology, Tehran University of Medical Sciences, Tehran, Iran

## Abstract

Spinal cord injury (SCI) is a debilitating condition for which no definitive treatment has yet been identified. Notably, it influences other tissues through inflammatory reactions and metabolic disturbances. Therefore, fingolimod (FTY-720), as an FDA-approved inflammatory modulator, would be promising. In the present study, nanocarriers with two distinct monodisperse particle sizes of 60 (nF60) and 190 (nF190) nm were prepared via low-(stirring) and high-energy (probe ultrasound) emulsion oil in water (O/W) methods. Larger nanocarriers showed higher EE% and sustained-release profile than smaller nanocarriers. Neural stem cell (NSC) viability and lactate dehydrogenase (LDH) release were studied in the presence of nanocarriers and free FTY-720. The results indicated that nanocarriers and free FTY-720 enhanced NSC viability compared with the control group. However, nF190 induced significantly less cell membrane damage than nF60. Nanocarriers and free FTY-720 enhanced motor neuron recovery in SCI rats, while body weight and return to bladder reflux by nF190 were significantly higher than those in the nF60 group. Return to bladder reflux might be due to the role of FTY-720 in the regulation of detrusor muscle tone and preservation of the integrity of vessels by acting on endothelial cells. Moreover, nF190 gained higher soleus muscle weight than the free drugs; probably decreasing proinflammatory cytokines in the soleus diminishes muscular atrophy in SCI rats. In summary, it might be said that larger nanocarriers with sustained-release profile and less cell membrane damage seem to be more efficient than smaller ones to manage SCI and enhance bladder reflux. These data will help pharmaceutical companies select the correct particle size for nanodrugs and develop more efficient drug formulations to treat SCI.

## 1. Introduction

Spinal cord injury (SCI) is a severe and debilitating condition that leads to a variety of complications, from transient neurologic impairment to permanent motor and sensory function loss [1]. According to the WHO, the annual incidence of SCI is between 250000 and 500000 cases worldwide [2]. The advancement of technology and the convergence of research disciplines have overcome many medical obstacles. However, the development of an efficient therapeutic approach for SCI is complicated and problematic due to the extensive axonal loss at the moment of injury and neuronal regeneration restriction of the human central nervous system [3]. However, it seems that hydrogel-based materials such as self-assembling peptide nanofibers are of interest [4–6]. The pathology of SCI is classified into primary and secondary injuries. Primary injury refers to a mechanical insult to axons, blood vessels, and the cell membrane at the moment of impact, and secondary injury is the subsequent neurodegenerative process leading to ischemia, inflammation, necrosis, apoptotic cell death, and glial scar formation [7]. The main focus of SCI treatment is to counteract the cascade of secondary injury mechanisms.

Methylprednisolone, a synthetic anti-inflammatory and immunosuppressive glucocorticoid, is the current gold standard for SCI patients. However, the safety and efficacy of this therapeutic agent have been subject to debate [8]. We proposed fingolimod (FTY-720), an immunosuppressant and anti-inflammatory small molecule, to treat SCI in the present study. FTY-720, as a nonselective sphingosine-1-phosphate (S1P) receptor modulator, is the first orally approved medication for relapsing-remitting multiple sclerosis (RRMS). It decreases the rate of relapse in RRMS patients by one-half. There is increasing evidence that FTY-720 may be helpful for neuronal reconstruction [9] and attenuating SCI. It has been disclosed that traumatic damage results in the release of neural self-antigens; therefore, immunomodulatory drugs to modulate immunological reactions following trauma are of interest [10]. In one study, Efstathopoulos et al. showed the ability of FTY-720 to induce adult mouse hippocampal neurogenesis [11]. In another study, PLGA/FTY-720 microfibers stimulated NSC differentiation into neurons and oligodendrocytes and suppressed astrocytosis [12]. A number of studies have reported that FTY-720 decreases T-cell infiltration and gliosis and enhances motor function recovery in an SCI rat model [10, 13]. Since S1P receptors are expressed in various kinds of cells, this S1P analog could affect different aspects of the secondary injury process. Norimatsu et al. proposed the immune-independent potential capability of this medicine on tissue preservation and functional recovery after SCI [13]. Likewise, Colombo et al. suggested that FTY-720 inhibits inflammation and glial scar formation through the blockade of NF-*κ*B translocation [14]. However, implantation of electrospun PLGA/FTY720 microfibers into a transaction rat model manifested increased functional recovery outcomes [12].

Medical nanotechnology strategies have provided significant breakthroughs over the past several decades. Nanoparticle formulations have been successfully employed to treat and ameliorate many diseases and disorders, including advanced cancer, diabetes, HIV, and cardiovascular disease [15]. A large surface area to mass ratio, enhanced bioavailability, prolonged retention, reduced toxicity, increased therapeutic efficacy, and biocompatibility are some benefits of nanodrug systems as an alternative to conventional drugs [15]. Nanoemulsions are heterogeneous colloidal dispersions consisting of a mixture of two immiscible liquids stabilized by amphiphilic surfactants. These lipid-based formulations are considered a kinetically stable system and can be prepared by employing low- and high-energy methods [16, 17]. Drug delivery with nanoemulsions is a simple yet effective method for encapsulating hydrophobic drugs.

Despite several investigations on the potential of nanocarriers for SCI recovery, we do not know which particle size would be effective in recovering spinal cord injury. These data will help pharmaceutical companies develop more efficient drug formulations to treat SCI. The present study responds to whether FTY-720 nanoemulsions enhance therapeutic efficacy compared to their bulk counterparts in a contusion SCI rat model. Meanwhile, it defines which particle size is more efficient for SCI recovery.

## 2. Methods

### 2.1. Preparation of Fingolimod-Loaded Nanoemulsion

FTY720 nanocarriers at two different particle sizes with equal concentrations of FTY-720, oil, surfactant, and cosurfactant were prepared via low (stirring) and high-energy (probe ultrasound) emulsion oil in water (O/W) methods [18]. In brief, a mixture of 1 mg/ml fingolimod, 2% (*w*/*w*) mineral oil, 6% (*w*/*w*) Span 80-Tween 80 (surfactant), 1% (*w*/*w*) ethanol (cosurfactant), and distilled water was exposed to either a magnetic stirrer (800 rpm, 10 min) and/or an ultrasound probe (400 W s^−1^, 4 min) to obtain 190 nm and 65 nm oil-in-water (o/w) fingolimod nanoemulsions. Nanoemulsions were then stored in sealed glass vials covered with aluminum foil for further investigation. In this paper, NF60 and NF190 will be referred to as fingolimod nanoemulsions with 65 nm and 190 nm particle sizes, respectively.

### 2.2. Nanoemulsion Characterization

#### 2.2.1. Particle Size and Zeta Potential

The hydrodynamic particle size and zeta potential of nanocarriers were studied using a dynamic light scattering (DLS) apparatus (Scatteroscope I, Qudix, South Korea and Malvern Instrument Ltd., UK) at a refractive index of 1.531 and neutral pH to avoid the impact of the false charge on the zeta potential. The assay was performed in triplicate, and the mean ± SD was reported.

#### 2.2.2. Morphological Analysis Using a Scanning Electron Microscope (SEM)

The surface morphology, shape, and size of the nanoparticles were evaluated using SEM (KYKY–EM3200, China). Before imaging, one droplet of nanocarrier was mounted on a glass slide and dried. Then, the samples were coated with gold, and SEM was recorded at 20 kV.

#### 2.2.3. Entrapment Efficacy Percentage (EE%)

Ultrafiltration is a gold method to evaluate nanocarriers' entrapment efficacy (EE). Indirect method was used to evaluate the amount of encapsulated drug. The newly synthesized nanocarriers in Amicon microtubes were centrifuged for 15 min at 14000 G. The supernatant that contained the unencapsulated drug was removed, and absorbance was read using RIGOL ULTRA 3660 spectrophotometer at a wavelength of 217 nm. EE was calculated using the following formula;

(1) $$\begin{array}{c} \left(C-\frac{\text{TC}}{C}\right)\times 100, \end{array}$$

where *C* is the total amount of FTY-720, and TC is the free amount of FTY-720, which was detected only in the supernatant media. The assay was performed in triplicate, and the values provided are the mean ± SD of three independent experiments.

#### 2.2.4. Drug Release Profile

Franz diffusion cell was used to investigate the release profile of FTY-720 nanocarriers. 1 ml of each nanoemulsion was placed on a dialysis bag at the receptor part of the Franz diffusion cell. Franz diffusion cells was filled with PBS solution. The receptor and sampling port were completely covered with parafilm. Franz diffusion cells were placed on a shaker at 37°C at 100 rpm for 48 hours. For sampling at different times, 1 ml of the solution is pipetted out of the sampling port and immediately replaced with 1 ml PBS, and the tube end is completely closed again with parafilm. Sampling was performed at interval times of 1, 10, 20, 30 min, 1 h, 2 hours, 4 hours, 24 hours, and 48 hours. The absorbance of the samples was read using a RIGOL Ultra 3660 spectrophotometer at a wavelength of 217 nm, and the accumulated release rate of the drug at different times was plotted by Excel.

### 2.3. Cell Viability Assay

Neural stem cells (NSCs) were isolated from the subventricular zone (SVZ) of the lateral ventricles and seeded in NPBM as a cell culture medium. To evaluate the cell viability of nanocarriers and bulk drug, an MTT assay was performed. NSCs were seeded in a 96-well plate (10^4^ cells/well) for 24 h, and then, FTY-720 and FTY-nanocarriers were added to NCSs at a concentration of 10 ng/ml for 48 h. The cell media was removed, and 100 *μ*l of 3-(4,5-dimethylthiazol-2-Yl)-2,5 diphenyltetrazolium bromide (Sigma, USA) (0.5 mg ml−1 PBS) was added to the triplicate wells at 37°C in 5% CO2 and 95% moisture for 4 h. DMSO was added, and after 20 min, the absorbance was read using an ELISA reader (Bio-Tek) at 570 nm. The assay was repeated three times in triplicate, and the mean ± SD was reported.

### 2.4. Lactate Dehydrogenase Release (LDH)

Isolated NSCs were treated with FTY-720, nF190, nF60, and the control group. After 24 h, 100 *μ*l of cell supernatant was transferred to a 96-well plate and mixed equally with an LDH solution kit (Roche). After 20 min, the absorbance was read using an ELISA reader (Bio-Tek) at 490 nm. The assay was repeated three times in triplicate, and the mean ± SD was reported.

### 2.5. Severe SCI Contusion Model

The Iranian Ethical Committee of Iran University of Medical Sciences approved all experimental protocols and animals used in this study (IR.IUMS.REC.1399.087). All procedures were performed in accordance with the Iranian Ethical Committee for Animal Care and use. The study was carried out in compliance with the ARRIVE guidelines. All experimental procedures were performed in accordance with the relevant guidelines and regulations. Acute severe SCI was induced in 24 male Wistar rats (220–250 g) using the weight compression method, with 6 rats in each group [19]. Rats were randomly and equally divided into four groups, including FTY-720, nF190, nF60, and the control (PBS) groups. Animals were intramuscularly (IM) anesthetized with ketamine/xylazine (80 mg/kg and 10 mg/kg). Complete thoracic laminectomy was performed at the T9 level, the exposed spinal cord was subjected to a contusion impactor, and a severe SCI model was induced. Following injury, 10 *μ*l of the nanocarriers, FTY-720, and PBS at a concentration of 10 ng/ml were injected using a 26 gauge Hamilton syringe at a speed of 1 *μ*l/min at the lesion epicenter. The muscles and skin were sutured, and the animals were kept on a heating path until they awoke. Animals were monitored constantly and maintained with free access to water and food. They received antibiotics (5% gentamicin) daily for five days postsurgery.

### 2.6. Behavioral Analysis

The Basso Beattie Bresnahan (BBB) locomotor open-field locomotor test was carried out to examine hind limb stepping movements at days 1, 7, 14, 21, 28, 35, and 42 postinjury. The rat was placed in a Plexiglas circular apparatus (107 cm diameter, 60 cm wall height) with a nonslip floor. BBB score assessment was performed by a portable camera for 4 min, evaluated by two blinded independent observers, and averaged from both hind limbs. The scores ranged from 0 to complete paralysis and 21 to normal locomotion.

### 2.7. Return of Bladder Reflux

After SCI, the sacral micturition center may send signals to the bladder to squeeze. Bladder emptying was performed twice a day manually until reflex function was regained. The regain of spontaneous bladder function was regarded as a measure of recovery. The mean ± SD was reported for the four groups.

### 2.8. Weight Gain Evaluation

Weight gain is a marker of recovery in SCI. Animals were weighed before surgery and at days 1, 7, 14, 21, 28, 35, and 42 postinjury. Then, weight gain was compared on the first day. The mean ± SD was reported for the four groups.

### 2.9. Weighting of the Gastrocnemius and Soleus Muscles

The soleus and gastrocnemius muscles are essential muscles in walking and running. Muscle atrophy is adjacent to less movement. Therefore, in this study, the weight of the soleus and gastrocnemius muscles was measured in rats on the 42^nd^post surgery. To dissect the soleus muscle, the skin was detached, and the Achilles tendon was removed. After lifting the gastrocnemius muscle, the underlying soleus muscle was exposed, and then both muscles were sectioned for weighing. The mean ± SD was reported for the four groups.

#### 2.9.1. Histological Assessments

On day 42 postinjury, rats were transcardially perfused with PBS and fixed with 4% paraformaldehyde in 0.1 M PBS. Spinal cords were isolated, and transverse sections with a thickness of 5 *μ*m were obtained from the paraffin-embedded spinal cords. Sample slides were stained with hematoxylin and eosin (H&E) and covered with coverslips. The camera captured images at a resolution of 40X.

### 2.10. Statistical Analysis

GraphPad Instat software version 3 was applied to analyze particle mean size, zeta potential, cell viability, body weight, muscle weight, and BBB scores. Data were reported as the mean ± SD. One-way ANOVA (analysis of variance) was used for statistical analysis. The significance level was set at a *p* value less than 0.05.

## 3. Results and Discussion Section

### 3.1. Nanocarrier Characteristics

One of the most challenging issues in pharmaceutics is defining an effective particle size to recover SCI. Recent decades have witnessed an explosive growth in the design and delivery of nanomedicine. In this regard, FTY nanocarriers with two distinct particle sizes were prepared and compared, and their therapeutic efficacy was investigated in an SCI rat model. We assumed that encapsulation of FTY-720 into a nanoemulsion drug delivery system probably promotes neuronal survival and functional reconstruction of this powerful immunomodulatory medicine.

DLS was performed to study the particle size and zeta potential of the stable nanocarriers. DLS results showed that the nanocarriers synthesized by stirring and ultrasound methods had particle sizes of 60 and 195.5 ± 7.78 nm, respectively (*p* < 0.001). Meanwhile, they showed that the monodisperse nF60 and nF190 nanocarriers had PDI values of 0.1 and 0.2, respectively (Figures 1(a) and 1(b)). In other words, the low-energy emulsification method produced larger nanocarriers than the high-energy methods of ultrasound. However, both methods with an optimized oil, surfactant, and cosurfactant ratio make monodisperse nanoemulsions.

*ζ*-Potential data related to nF60 and nF190 showed a slightly negative surface charge. The *ζ*-potentials of the nF60 and nF190 nanocarriers were −9.98 ± 0.15 mV and −10.58 ± 0.35 mV, respectively. Their *ζ*-potentials were significantly different (*p* = 0.0198). Smaller nanocarriers showed less negative *ζ*-potential than larger nanocarriers. However, both showed *ζ*-potentials of approximately -10 mV.

SEM micrographs revealed that both the nF60 and nF190 nanocarriers had spherical morphology with uniform size and homogeneous distribution without agglomeration (Figures 1(c)–1(e)). Environmental conditions such as temperature and ionic strength influence the curvature of a polar spontaneous nanoemulsions. It might be said that the heating produced by the ultrasound method reduces the particle size of nanocarriers to more homogeneous particles (PDI: 0.1) by decreasing the viscosity and interfacial tension between the oil and water phases. However, cooling following the high energy method reduces the particle velocity and enhances the oil phase viscosity [20].

### 3.2. Entrapment Efficiency Percentage (EE%)

The EE% was measured using the ultrafiltration method. Results showed NF190 had higher EE% (83.42% ± 1.22) than NF60 (65.98% ± 1.82). There was significant difference between the EE% of both nanocarriers (*p* < 0.0002). Larger nanocarriers had higher capacity to entrap the FTY-720.

### 3.3. Drug Release Profile of Nanocarriers

The drug release profile of nanocarriers was evaluated using Franz diffusion cell. Statistical analysis of drug release showed that in the first four hours of drug release, both drugs had a high velocity slope and nonsignificant difference (*p* > 0.05). After 24 hours, the release rate of the two drugs was different (*p* < 0.001). This difference continued until the second day and at the end of 48 hours, and the release slope of the NF190 was lower than the release slope of the NF60 (*p* < 0.001). After 48 hours, in the larger sample, the accumulated release rate was 55% and in the smaller sample, and the accumulated release rate was 74% (*p* < 0.001). Larger nanocarriers that had higher EE% released FTY-720 in slower rate and more sustained-release profile than smaller nanocarriers (Figure 2).

### 3.4. NSC Viability and LDH Release

NSC viability was evaluated in the face of the nanocarriers and FTY-720 at a concentration of 10 ng/ml. The results indicated that there was no significant difference between the cell viability of nanocarriers together and compared to the bulk drug (*p* > 0.05). However, the control group had significantly less cell viability than the nanocarriers and bulk FTY-720 (*p* < 0.001). Nevertheless, both nanoemulsions manifested higher cell viability compared to the control group. It seems that FTY-720 can significantly enhance NSC viability and may be considered a promising drug for neurogenesis (Figure 3(a)). Zhang et al. [21] reported that FTY-720 at a concentration of less than 5 nM was more efficient than 10 nM in differentiating NSC to mature oligodendrocytes and decreasing GFAP as a marker of reactive astrocytes. Moreover, TUNEL-positive cells treated with FTY-720 at the concentrations of 0.1 to 10 nM were dose-dependent and showed more TUNEL-positive cells at the concentration of 5 and 10 nM. FTY-720 increases cell proliferation in part through S1P5/ERK [21, 22] and sonic hedgehog (Shh) signaling pathways [23]. Although FTY-720 at higher concentrations turns NSC into neural cells, NSC is more viable at lower concentrations of 5 nM. This is a reason for lower cell membrane damage in NSCs treated with nF190. The first point is the effect of FTY-720 on cell viability that is dose-dependent, and it has more biocompatible for neurons in less concentration. The second point is that release of FTY-720 from nF190 is slower and in a sustained-release manner than the nF60. Therefore, it might be postulated that FTY-720 nanocarriers that release less FTY-720 during a specific time interval (nF190) and in a more extended period are more biocompatible to neurons and less cytotoxic to damage cell membrane and release LDH.

There is just one report belonging to our group associated with the dependency of neurotoxicity on drug nanocarrier particle size. There are some other reports related to the effect of nanocarriers on different cell types, such as fibroblasts. For example, mesoporous silica NPs with a particle size of 250 nm induced higher endothelial toxicity than 30 nm NPs in part through the mitophagy mechanism [24]. Moreover, Tavakol et al. reported that larger curcumin nanocarriers induce higher fibroblast cell viability than smaller nanocarriers with a particle size of approximately 60 nm through the downregulation of Bax and NF*κ*B genes [25].

Earlier, we showed that small nanocarriers exhibited higher cellular viability than larger nanocarriers in neural BE (2)-M17 cells. These data are contrary to our recent results and are due to different cell types. Therefore, in neurotoxicity investigations, the cell type is critical, and we cannot refer to an outcome to other cell types. Although nanocarriers with a particle size of 60 nm may be considered a candidate particle size in dopaminergic cells, larger nanocarriers of 190 nm will act as the preferred particle size for SCI recovery. In addition, silica NPs in the range of 200 nm exhibit significantly higher neuronal viability than small NPs (50 nm) through calcium perturbation and apoptosis mechanisms [26]. However, in accordance with our results, Prabhu et al. demonstrated that copper NPs with particle sizes of 40, 60, and 80 nm did not induce a significant impact on the cell viability of DRG neurons [27]. In addition, Coelho et al. reported the antiapoptosis mechanism of FTY-720 to enhance oligodendrocyte viability [28]. These data were similar to our study in that FTY-720 increased neural cell viability compared to the control group.

To further study the effect of nanocarriers and bulk FTY-720 on NSCs, LDH release as a marker of necrosis and cell membrane damage was investigated. The results showed that smaller nanocarriers exhibited more serious cell membrane damage to NSCs and produced higher LDH release than larger nanocarriers (*p* < 0.01). At the same time, there was no significant difference between the other groups (*p* > 0.05). In other words, it seems that larger nanocarriers induced minor NSC membrane damage, while there was no significant difference between the cell membrane damage of smaller nanocarriers and bulk FTY-720 (*p* > 0.05) (Figure 3(b)). In summary, it seems that although both nanocarriers induced significantly high cell viability in NSCs, smaller nanocarriers caused higher NSC membrane damage compared to the larger nanocarriers with 190 nm particle size. Prabhu et al. disclosed that small and large copper NPs of 40 and 80 nm did not significantly induce LDH release from DRG neurons, and notably, these NPs significantly induced higher LDH release compared to the control group [27]. Moreover, Gillespie et al. reported that although both fine and ultrafine particles induced apoptosis in neural cells, ultrafine particles induced more apoptosis of neural cells than fine particles [29]. This finding was in good agreement with our results that larger nanocarriers induced less cell membrane damage of NSCs.

### 3.5. BBB Score

Nanocarriers and FTY-720 were directly injected into the lesion to investigate their effects on the SCI model. In vivo SCI models were exerted on Wistar male rats employing the weight drop contusion model. Blunt injury models, including weight drop, represent human injuries and can efficiently study secondary damage [3]. Herein, we chose local administration to transport the medicine across the blood-spinal cord barrier directly to the lesion area. Local delivery significantly decreases systemic administration side effects and effectively eliminates the risk of potential exposure and toxicity within the nontargeted organs [15].

To assess motor function recovery, BBB open-field locomotor rating scales were carried out in contusion rat models that received local FTY- nanocarriers and bulk drug for six weeks postinjury (Figure 3(c)). In the first four weeks, no significant difference was detected among the different groups. However, from week four, nanocarriers and bulk FTY-720 started to show a gradual rise in BBB score compared to the control group. Finally, bulk FTY720 and nanocarriers induced improved motor hind limb function compared to the control group (*p* < 0.001). There was no significant difference between the motor neuron recovery of nanocarriers and free FTY-720 (*p* > 0.05). These findings were in accordance with the MTT assay data. It seems that NSC viability has a direct impact on the potential of nanocarriers to enhance motor neuron recovery. To further investigate the effect of nanocarriers on SCI rats, bladder reflux and body and muscle weights were evaluated.

### 3.6. Return of Bladder Reflex

Impaired bladder function is another incapacitating consequence of SCI in humans and animals. The degree of SCI severity is correlated with bladder dysfunction [10]. In other words, the return of the bladder reflex was considered a sign of improvement and recovery. As shown in Figure 4(a), nF190 nanocarriers exhibited a noticeably faster regain of spontaneous bladder function compared to nF60 (*p* < 0.01), free drug (*p* < 0.05), and the control group (*p* < 0.001). There was no significant difference between the return of bladder reflux in the nF60 and free drug groups (*p* > 0.05). Probably, the more sustain and longer release profile of NF190 resulted in quicker return of bladder reflux. Based on these results, although larger nanocarriers could enhance motor neuron recovery at the nF60 and free drug scores, they positively impacted bladder reflux, which is very important in SCI patients. Lee et al. demonstrated that daily IP injections of FTY-720 for four weeks following a contusion model in a Long-Evans hooded rat model significantly enhanced functional outcomes and bladder recovery [10]. Moreover, FTY-720 regulates detrusor muscle tone and preserves the integrity of vessels by acting on endothelial cells [30].

### 3.7. Body Weight Change

Body weight changes were recorded weekly as an indicator of general health and recovery [10]. The weight of the animals was recorded each week until sacrifice (Figure 4(b)). There was a marked decline in body weight in all groups in the first week after surgery. All animal weights increased over time, as expected. However, this increasing trend was more significant in the nanocarrier-treated groups (*p* < 0.001). By the time, the body weight of rats treated with nanocarriers was significantly enhanced compared to the control group and free drug at four weeks. nF190 induced significantly higher body weight than nF60 at 42 days posttreatment (*p* < 0.001).

Meanwhile, nF60 significantly influenced higher body weight than the free drug (*p* < 0.001). Based on these findings, it seems that although there was no significant difference in motor neuron recovery of nanocarriers and free drugs, gained body weight and bladder reflux, as markers of health and recovery in rats, were enhanced using nF190 and nF60. Eventually, the return of the bladder reflex in SCI rats positively impacted body weight and general recovery.

### 3.8. Gastrocnemius and Soleus Muscle Mass

Skeletal muscle is an endocrine organ [19] associated with inflammation. Therefore, inflammation leads to muscle atrophy and reduced satellite cells [31, 32]. Muscle atrophy leads to metabolic disorders in SCI patients [33]. In this study, the gastrocnemius and soleus muscles were dissected and weighed after perfusion on the 42^nd^ day. The results showed no significant difference between the gastrocnemius weights of the groups (*p* = 0.0982). There is some difference between the two types of gastrocnemius and soleus muscles, in which the gastrocnemius is predominantly glycolytic muscle while the soleus is more largely slow-twitch muscle [34]. At the same time, soleus muscle mass was higher in the nF190 (*p* < 0.01) and nF60 (*p* < 0.05) groups than in the control group. nF190 showed significantly higher soleus weight than the free drug (*p* < 0.05) (Figure 4(c)). Probably, higher EE% of larger nanocarriers along with its more sustain and longer release profile resulted in higher recovery of soleus muscle mass compared to smaller nanocarrier. Fingolimod can influence in longer period on neural and muscle tissues. Based on these findings, it might be said that larger nanocarriers can diminish soleus muscle atrophy. Ormond et al. showed that greater soleus muscle weight is correlated with better hind limb functional recovery [35]. Watterson et al. showed a regulatory effect of FTY720 on detrusor muscle tone in a rabbit model [36]. Graham et al. showed that SCI induces the upregulation of IL-6, TNF*α*, and p53 in soleus muscle, while IL-6 and TNF*α* return to baseline in a short period [34]. However, the return of inflammatory cytokines to baseline occurs in rodents [37], and they cannot undergo senescence and may not translate to humans. In other words, in humans, inflammatory cytokines following SCI promote cellular senescence in muscle. Since FTY-720 reduces the upregulation of proinflammatory cytokines such as IL-17A, IL-1, IL-6, and TNF*α* [33, 38, 39], nF190 diminished soleus muscular atrophy in SCI rats.

### 3.9. Histological Evaluation

Histological evaluation was performed using H&E staining. As demonstrated in Figure 4, a scar was made in the spinal cord adjacent to the T9 spine in this model. In the control group, the cavity was significantly larger and more extended outside than in the other groups on the 42^nd^day posttreatment. At the same time, the cavity had a smaller size in nF190. Since a severe model was induced in the spinal cord, the astroglial scar could not completely recover in all groups, and fibroconnective tissue was observed in the cavity of all groups. However, the nanocarriers showed less cavity size compared to others. It seems that nanocarriers help the astroglial scar to be reconstructed (Figure 5).

Analyzing the functional recovery of SCI rats treated with free FTY-720, nF60, and nF190 indicated that nF190 remarkably improved the outcomes of faster regain of bladder reflux, gain of body weight, and soleus muscle compared to free FTY-720 and in some parts more than smaller nanocarriers. Kong et al. discovered that PLGA microfibers containing FTY-720 and NSCs reduce the glial scar cavity size, suppress astrocyte differentiation, and induce NSC differentiation into neuron oligodendrocytes, which are critical for axonal reconstruction. The in vivo results of that study pointed out the remarkable efficacy of FTY-720 loaded into electrospun fibers on motor recovery in a spinal cord transection rat model [12]. Moreover, Norimatsu et al. demonstrated that FTY-720 has a more extensive activity than S1P1 receptor antagonists. They declared that permanent internalization of the S1P1 receptor in astrocytes through functional antagonism is probably a primary function for FTY-720 efficacy [13]. Although FTY-720 decreased the migration of lymphocytes to the site of SCI, it could not diminish the number of infiltrated granulocytes and glial cells [2]. Cytokines and other biomolecules released by these cells are in part responsible for the neurotoxicity of SCI. However, microglial scavenger debris and inhibitory biomolecules in SCI [40] help recover injured neurons through axon regeneration signaling [41]. Therefore, it seems that SCI recovery following SCI occurs in part through T-cell attenuation.

## 4. Conclusion

The high-energy method using an ultrasonicator and the low-energy method using a magnetic stirrer were employed to synthesize nanoemulsions with 60 and 190 nm particle sizes, respectively. Particle size was analyzed using SEM and DLS. Nanocarriers were biocompatible and exhibited higher cell viability than the control group. Local delivery of the FTY-720 nanoemulsion after the contusion model in an SCI rat model significantly improved hindlimb motor function recovery. Collectively, our data demonstrated that nF190 provides us with neuroprotective and neuroregenerative properties. This synthetic nanocarrier not only impedes further damage but also helps to improve motor dysfunction and recovery. Nanocarriers at a particle size of 190 nm through higher EE%, sustained-release profile of FTY-720 that releases less amount of FTY-720 during a specific time interval, enhanced cellular uptake positively impact bladder reflex, bodyweight, and muscular weight. Eventually, smaller nanocarriers through enhanced cell membrane damage than nF190 exhibit less beneficial effects than nF60 in SCI rats. The results of the presented investigation not only are important for pharmaceutical companies as a view of neurosurvival but also are valuable to select the favorable particle size in the treatment of spinal cord injury. It might be said that not only body weight and return to bladder reflux by larger nanocarriers was significantly higher than smaller nanocarriers but also larger nanocarriers promoted higher recovery of spinal cord injury. We suggest that nanocarriers can be studied in a moderate SCI model to significantly show the impact of particle size on motor neuron recovery.

## Figures and Tables

**Figure 1:** Characterization of nanocarriers using (a, b) DLS and (c, d) SEM. DLS graph of (a) ~190 nm and (b) 60 nm particles, and SEM micrographs of (c) ~190 nm and (d) 60 nm particles showed that nanocarriers with uniform size were dispersed in water (e) shows particle size distribution of nanocarriers acquired by SEM.

**Figure 2:** Release profile of FTY-720 from nanocarriers. ^∗∗∗^ indicated *p* < 0.001.

**Figure 3:** (a) Cell viability percentage of NSCs treated with nF60, nF190, and bulk FTY-720 at 10 ng/ml concentrations for 48 h. The control group showed significantly less NSC viability than the other groups. (b) LDH release from NSCs treated with nF60, nF190, and bulk FTY-720 at 10 ng/ml concentrations for 24 h. nF190 showed significantly less LDH release from NSCs than nF60. (c) BBB rating scale in the severe SCI model that received NF60, NF190, bulk fingolimod, and PBS (control) at days 1, 7, 14, 28, 35, and 42 postinjury by two blinded observers. NF190 showed a significantly higher functional recovery score than the other groups (^∗^*p* < 0.05, ^∗∗^*p* < 0.01, and ^∗∗∗^*p* < 0.001). ^∗^ indicates *p* < 0.05, ^∗∗^ indicates *p* < 0.01, and ^∗∗∗^ indicates *p* < 0.001.

**Figure 4:** (a) On the first day of regaining normal bladder function, SCI rats received nF60, nF190, free FTY-720, and PBS to the legion area. Normal bladder expression was restored in all animals within 10 days. nF190-treated rats were the first group to regain spontaneous bladder function. (b) The body weight of SCI rats was monitored 42 days postinjury. In the first week following SCI, all groups experienced considerable weight loss. Animals that received nF190 showed promoted body weight gain on day 42. (c) Soleus and gastrocnemius muscles were weighed in severe model SCI rats treated with nF60, nF190, free FTY-720, and PBS after perfusion. nF190 showed improved soleus muscle weight compared with free drug and control groups. (^∗^ indicates *p* < 0.05, ^∗∗^ indicates *p* < 0.01, and ^∗∗∗^ indicates *p* < 0.001).

**Figure 5:** Histological H&E staining of injured spinal cord in rats on day 42. As shown in the captured image, the cavity could not completely recover in all groups, and nF190 showed a stronger recovery effect than the other groups (X40, scale bar = 20 *μ*m). SC means astroglial scar, and RG means regenerated tissue.

## Data Availability

The data that support the findings of this study are available upon reasonable request from the authors.

## Additional Points

*Preprint*. A preprint has previously been published on Research Square [42]“Under Reference: [42] according to the following link: https://assets.researchsquare.com/files/rs-530238/v1/317ef7a9-3c90-4849-bc1e-dc6a2cf1f37e.pdf?c=1635226151. Delaram Poormoghadam Bita Rasoulian Shiadeh Fereshte Azedi Hani Tavakol Seyed Mahdi Rezayat Shima Tavakol Particle Size of Drug Nanocarriers Defines the Fate of Spinal Cord Injury's Recovery. doi:10.21203/rs.3.rs-530238/v1.

## References

[1] Ahuja C. S., Wilson J. R., Nori S. (2017). Traumatic spinal cord injury. *Nature reviews Disease primers*.

[2] https://www.who.int/news-room/fact-sheets/detail/spinal-cord-injury.

[3] Kwon B. K., Tetzlaff W., Grauer J. N., Beiner J., Vaccaro A. R. (2004). Pathophysiology and pharmacologic treatment of acute spinal cord injury. *The spine journal*.

[4] Tavakol S., Saber R., Hoveizi E., Aligholi H., Ai J., Rezayat S. M. (2016). Chimeric self-assembling nanofiber containing bone marrow homing peptide’s motif induces motor neuron recovery in animal model of chronic spinal cord injury; an in vitro and in vivo investigation. *Molecular Neurobiology*.

[5] Tavakol S., Mousavi S. M. M., Tavakol B., Hoveizi E., Ai J., Sorkhabadi S. M. R. (2017). Mechano-transduction signals derived from self-assembling peptide nanofibers containing long motif of laminin influence neurogenesis in in-vitro and in-vivo. *Molecular Neurobiology*.

[6] Tavakol S., Musavi S. M. M., Tavakol B., Hoveizi E., Ai J., Rezayat S. M. (2017). Noggin along with a self-assembling peptide nanofiber containing long motif of laminin induces tyrosine hydroxylase gene expression. *Molecular Neurobiology*.

[7] Rogers W. K., Todd M. (2016). Acute spinal cord injury. *Best Practice & Research Clinical Anaesthesiology*.

[8] Wu W., Lee S.-Y., Wu X. (2014). Neuroprotective ferulic acid (FA)-glycol chitosan (GC) nanoparticles for functional restoration of traumatically injured spinal cord. *Biomaterials*.

[9] Tavakol S., Hoveizi E., Tavakol B. (2019). Small molecule of sphingosine as a rescue of dopaminergic cells: a cell therapy approach in neurodegenerative diseases therapeutics. *Journal of cellular physiology*.

[10] Lee K. D., Chow W. N., Sato-Bigbee C. (2009). FTY720 reduces inflammation and promotes functional recovery after spinal cord injury. *Journal of Neurotrauma*.

[11] Efstathopoulos P., Kourgiantaki A., Karali K. (2015). Fingolimod induces neurogenesis in adult mouse hippocampus and improves contextual fear memory. *Translational Psychiatry*.

[12] Kong W., Qi Z., Xia P. (2019). Local delivery of FTY720 and NSCs on electrospun PLGA scaffolds improves functional recovery after spinal cord injury. *RSC advances*.

[13] Norimatsu Y., Ohmori T., Kimura A. (2012). FTY720 improves functional recovery after spinal cord injury by primarily nonimmunomodulatory mechanisms. *The American journal of pathology*.

[14] Colombo E., di Dario M., Capitolo E. (2014). Fingolimod may support neuroprotection via blockade of astrocyte nitric oxide. *Annals of Neurology*.

[15] Braddock M. (2016). *Nanomedicines: Design, Delivery and Detection*.

[16] Karami Z., Zanjani M. R. S., Hamidi M. (2019). Nanoemulsions in CNS drug delivery: recent developments, impacts and challenges. *Drug Discovery Today*.

[17] Kumar M., Bishnoi R. S., Shukla A. K., Jain C. P. (2019). Techniques for formulation of nanoemulsion drug delivery system: a review. *Preventive nutrition and food science*.

[18] Poormoghadam D., Almasi A., Ashrafizadeh M., Vishkaei A. S., Rezayat S. M., Tavakol S. (2020). The particle size of drug nanocarriers dictates the fate of neurons; critical points in neurological therapeutics. *Nanotechnology*.

[19] Pedersen B. K., Febbraio M. A. (2012). Muscles, exercise and obesity: skeletal muscle as a secretory organ. *Nature Reviews Endocrinology*.

[20] Santana R., Perrechil F., Cunha R. (2013). High- and low-energy emulsifications for food applications: a focus on process parameters. *Food Engineering Reviews*.

[21] Zhang Y., Li X., Ciric B. (2017). Effect of fingolimod on neural stem cells: a novel mechanism and broadened application for neural repair. *Molecular Therapy*.

[22] Tan B., Luo Z., Yue Y. (2016). Effects of FTY720 (fingolimod) on proliferation, differentiation, and migration of brain-derived neural stem cells. *Stem cells international*.

[23] Zhang J., Zhang Z. G., Li Y. (2015). Fingolimod treatment promotes proliferation and differentiation of oligodendrocyte progenitor cells in mice with experimental autoimmune encephalomyelitis. *Neurobiology of Disease*.

[24] Orlando A., Cazzaniga E., Tringali M. (2017). Mesoporous silica nanoparticles trigger mitophagy in endothelial cells and perturb neuronal network activity in a size- and time-dependent manner. *International Journal of Nanomedicine*.

[25] Tavakol S., Zare S., Hoveizi E., Tavakol B., Rezayat S. M. (2019). The impact of the particle size of curcumin nanocarriers and the ethanol on beta_1-integrin overexpression in fibroblasts: a regenerative pharmaceutical approach in skin repair and anti-aging formulations. *DARU Journal of Pharmaceutical Sciences*.

[26] Ariano P., Zamburlin P., Gilardino A. (2011). Interaction of spherical silica nanoparticles with neuronal cells: size- dependent toxicity and perturbation of calcium homeostasis. *Small*.

[27] Prabhu B. M., Ali S. F., Murdock R. C., Hussain S. M., Srivatsan M. (2010). Copper nanoparticles exert size and concentration dependent toxicity on somatosensory neurons of rat. *Nanotoxicology*.

[28] Coelho R. P., Payne S. G., Bittman R., Spiegel S., Sato-Bigbee C. (2007). The immunomodulator FTY720 has a direct cytoprotective effect in oligodendrocyte progenitors. *Journal of Pharmacology and Experimental Therapeutics*.

[29] Gillespie P., Tajuba J., Lippmann M., Chen L.-C., Veronesi B. (2013). Particulate matter neurotoxicity in culture is size-dependent. *Neurotoxicology*.

[30] Brinkmann V., Cyster J. G., Hla T. (2004). FTY720: sphingosine 1-phosphate receptor-1 in the control of lymphocyte egress and endothelial barrier function. *American Journal of Transplantation*.

[31] Londhe P., Guttridge D. C. (2015). Inflammation induced loss of skeletal muscle. *Bone*.

[32] Verdijk L. B., Dirks M. L., Snijders T. (2012). Reduced satellite cell numbers with spinal cord injury and aging in humans. *Medicine and science in sports and exercise*.

[33] Luo Y.-T., Liang Y.-F., He H., Zhang M.-T., Wang R., Li H.-L. (2020). The immunosuppressant fingolimod ameliorates experimental autoimmune myasthenia gravis by regulating T-cell balance and cytokine secretion. *American journal of translational research*.

[34] Graham Z. A., Goldberger A., Azulai D. (2020). Contusion spinal cord injury upregulates p53 protein expression in rat soleus muscle at multiple timepoints but not key senescence cytokines. *Physiological Reports*.

[35] Ormond D. R., Shannon C., Oppenheim J. (2014). Stem cell therapy and curcumin synergistically enhance recovery from spinal cord injury. *PLoS One*.

[36] Watterson K. R., Berg K. M., Kapitonov D. (2007). Sphingosine-1-phosphate and the immunosuppressant, FTY720-phosphate, regulate detrusor muscle tone. *The FASEB Journal*.

[37] Phillips E. G., Beggs L. A., Ye F. (2018). Effects of pharmacologic sclerostin inhibition or testosterone administration on soleus muscle atrophy in rodents after spinal cord injury. *PLoS One*.

[38] Thomas K., Sehr T., Proschmann U., Rodriguez-Leal F. A., Haase R., Ziemssen T. (2017). Fingolimod additionally acts as immunomodulator focused on the innate immune system beyond its prominent effects on lymphocyte recirculation. *Journal of Neuroinflammation*.

[39] Yu H., Herbert B. A., Valerio M., Yarborough L., Hsu L.-C., Argraves K. M. (2015). FTY720 inhibited proinflammatory cytokine release and osteoclastogenesis induced by Aggregatibacter actinomycetemcomitans. *Lipids in health and disease*.

[40] Banati R. B., Graeber M. B. (2004). Surveillance, intervention and cytotoxicity: is there a protective role of microglia?. *Developmental neuroscience*.

[41] Yin Y., Henzl M. T., Lorber B. (2006). Oncomodulin is a macrophage-derived signal for axon regeneration in retinal ganglion cells. *Nature neuroscience*.

[42] Poormoghadam D., Shiadeh B. R., Azedi F., Tavakol H., Rezayat S. M., Tavakol S. (2021). *Particle size of drug nanocarriers defines the fate of spinal cord injury’s recovery*.

